RETRACTED

# Construction of the Reverse Resource Recovery System of e-Waste Based on DLRNN

**DOI:** 10.1155/2021/2143235

**Published:** 2021-09-23

**Authors:** Changru Li

**Affiliations:** School of Public Administration, Hohai University, Focheng West Road, Nanjing 211100, China

## Abstract

The research on the reverse resource network of e-waste at home and abroad is still in its infancy, and most of it is only based on traditional forward logistics. Reverse resources are the process of moving goods from their typical final destination for recycling value or proper disposal. With the intensification of market competition and the strengthening of environmental protection legislation by the government, reverse resources are no longer a neglected corner in the supply chain. The DLRNN model of the e-waste reverse resource recovery system constructed in this paper can provide an important theoretical and empirical basis for the rational utilization of waste electronic products and fully tap the potential value of waste electronic products, which is of great significance to the recycling of natural resources. In this paper, a hybrid network framework DLRNN based on deep learning (DL) and cyclic neural network (RNN) is designed for problem classification. Experimental results show that the classification accuracy of this framework is improved by 2.4% on TREC and 2.5% on MSQC without additional word vector conversion tools.

## 1. Introduction

Due to the rapid development of the technology level of the electronic industry and the ever-expanding demand of the society for electronic consumer products, the electronic products are eliminated and updated very quickly, resulting in a large number of wastes, including all kinds of discarded computers, printers, communication equipment, household appliances, and precision electronic instruments and meters. The report on e-waste published by the European Union points out that this kind of e-waste increases by 16%–28% every five years, which is three times faster than other wastes [1]. Electronic waste contains a variety of dangerous and harmful substances; the main pollution components include lead, nickel, cadmium, mercury, hexavalent chromium, and brominated flame retardants. If these substances are not handled properly, they will have a great impact on the environment and human health [2, 3]. However, the resource characteristics of electronic waste are outstanding. If properly handled, it can not only effectively solve the problem of environmental pollution but also save a lot of resources and create considerable economic benefits [4]. Among them, the value of precious metals accounts for about 40%–70% of the total value of electronic wastes, which has an extremely high recycling value [5, 6].

RETRACTED

Due to political, economic, and cultural reasons, the recovery rate of electronic waste in China is very low, and the industrialization and scale of electronic waste recovery and treatment have not yet been realized. At present, the recycling, treatment, and disposal of electronic waste in China are mainly informal recycling channels [7]. The existing recycling system of electronic waste in China has scattered recycling channels, primitive treatment methods, and low value-added products. In addition to the inflow of a large number of foreign electronic wastes, as far as China is concerned, once electronic and electrical products become wastes, there are often four main destinations: the holders of electronic wastes store them themselves and enter the second-hand market, the individual recyclers dismantle them after purchasing them, and the recycling plants recycle them [8]. In this case, it is necessary to analyze the emergence and development of reverse resources of e-waste from the perspective of economics, conduct in-depth research, and grasp on the nature of its emergence and development, so as to promote the development of reverse resources of e-waste in China and keep it consistent with the circular economy goal of building a harmonious society [9, 10].

Deep learning (DL) is a technique that uses neural networks with no less than two hidden layers to perform nonlinear transformation or representation learning on input. Using the recurrent neural network (RNN) to extract and train data features will greatly reduce the sensitivity of DL to data samples. RNNDL algorithm is an artificial neural network which uses multiple single nodes to generate directional input and output connected into a ring. It transmits information in the flow of time and can use internal memory to process time series signals, but it cannot keep long-term memory, and can only remember information in a short time [11]. Based on this, this paper makes use of qualitative analysis and quantitative analysis, regards discarded mobile phones as the representative of e-waste, studies the corresponding network design for reverse resource network, and puts forward a construction method of reverse resource recovery system of e-waste based on DLRNN combined with DL and RNN.

## 2. Related Work

The characteristics of e-waste are as follows: (1) the growth momentum is very fast, and the waste of resources is caused; (2) garbage cannot be effectively recovered and reused, which brings serious harm to the environment; and (3) it also could bring serious harm to human health. The study in [12] pointed out that reverse resource is a broad term used to describe the logistics management and disposal of various harmful or harmless wastes from packaging to products, which includes reverse distribution that causes goods and information to flow in the opposite direction of normal logistics activities. The study in [13] found that the first person who is different from the forward logistics network, especially the location of the recycling center, especially the distributor, needs to accept many and scattered logistics sources, and its location is characterized by “many to few” or even “many to one,” and the traditional facility location model has been improved and perfected. The study in [14] summarized some basic characteristics of the reverse resource network system, including high complexity of network, complex diversity of targets, imbalance between supply and demand, and “from more to less” characteristics. This paper systematically and comprehensively analyzes the basic characteristics of the reverse resource network system, which lays a foundation for future research and development [15]. Aiming at the recycling system of used mobile phones in Britain, the current mainstream recycling network framework in Britain is constructed from three aspects: product flow, information flow, and incentive measures. The study in [16] analyzed and studied the mobile phone recycling systems of mobile phone manufacturers, mobile phone service providers, and mobile phone retail stores in the US market and summed up the differences in the structure of used mobile phone recycling networks between the US and Brazil. The study in [17] analyzed and studied two different reverse resource recovery modes—integrated and decentralized—and concluded that the decentralized mode is the best choice of reverse resource recovery mode. The study in [18] put forward that “return logistics is called reverse resources, with the purpose of effectively implementing product recovery,” and return products refer to products that have been used by consumers and abandoned in the forward supply chain and ended their life cycle. This definition involves the product life cycle theory.

RETRACTED

Reverse resource recovery is a series of activities and processes such as planning, executing, and controlling the WIP, inventory, finished products, and the corresponding information flow and capital flow from the end consumer to the initial source of supply, with the goal of properly treating the products or restoring part of their value. Reverse logistics is essentially a circular economy, which is an economic development model with the core of efficient utilization and recycling of resources; the basic characteristics of low consumption, low emission, and high efficiency; and the goal of sustainable development. In essence, the recycling process of electronic waste is to transfer it from consumers to producers as raw materials of new products, which is just opposite to the process of new products from producers to consumers, so it is also called reverse resources. The study in [19] studied the problem of the reverse resource network structure of waste electronic products and established mathematical programming models from the perspectives of owners, collectors, and material handlers of waste electronic products, and all parties take actions according to the principle of maximizing profits. The study in [20], aiming at the problems in the development of the reverse resource network in China's manufacturing enterprises, analyzed and studied by using the theory of circular economy; at the same time referred to the development models in the field of reverse resources at home and abroad; and put forward a series of constructive suggestions for the long-term development, technological development, and measures development of China's reverse resource industry. The study in [21] introduced the domestic and foreign problems about the recovery of municipal solid waste, including treatment technology and treatment methods, and made comparative analysis according to different treatment methods. Literature [22] divided the reverse resource network into recovery, inspection, reprocessing, resale, and waste disposal. According to different recycling methods of waste, the reverse resource network structure is divided into reuse, remanufacturing, recycling, and commercial return. The study in [23] analyzed the operation mode of reverse resource network recycling for waste electronic products at home and abroad and, on this basis, designed a new mode of reverse resource network recycling with recycling alliance as the main body. Literature [24] held that the government plays an important role in establishing and operating the reverse resources of waste electronic and electrical products.

To sum up, by consulting the relevant research literature at home and abroad, we can find that, in most of the literature, the setting condition of reverse resource network is the operation process in a deterministic environment. However, the uncertainty of reverse resources is much higher than that of the forward logistics and, in the actual operation of reverse resources, the amount of recycling, the number of nodes, and the amount of logistics between nodes are also uncertain, so the current literature has no practical significance in actual operation.

## 3. Research Method

### 3.1. Deep Learning

DL is machine learning aiming at building a deep structured model. Generally, it is agreed that the model contains at least three hidden layers. This kind of network with a multi-hidden-layer structure is difficult to be trained by common neural network algorithms, such as BP algorithm, because of the large amount of sample data and slow training process, and the parameters are easy to converge to the local rather than the global optimum, which is of little practical significance.

RETRACTED

The restricted Boltzmann machine (RBM) is an improvement on the Boltzmann machine [25]. The Boltzmann machine is a random network. Because of the interconnection between the units in its layer, the network training process is very slow. In 1986, Somlensky introduced a restricted Boltzmann machine, which includes an obvious layer and a hidden layer, and there is no interconnection between the units in the layer. Therefore, it becomes very efficient to use RBM for reasoning calculation.

Assuming that an RBM contains *n* visual units and *m* hidden units, the states of visual units and hidden units may be represented by vectors *v* and *h*, where *v*_*i*_ represents the state of the *i*th visual unit and *h*_*j*_ represents the state of the *j*th hidden unit. Then, for a given set of states *v* and *h*, the joint probability distribution of RBM as a system can be expressed by energy function:

(1) $$\begin{array}{c} E\left(v,h\right)=-\sum_{i=1}\sum_{j=1}^{m}W_{ij}v_{i}h_{j}-\sum_{i=1}^{n}v_{i}b_{i}-\sum_{j=1}^{m}h_{j}c_{j}. \end{array}$$

Here, *W*_*ij*_, *c*_*i*_ is the parameter of RBM. *W*_*ij*_ represents the connection strength between the visual unit *i* and the hidden unit *j*, *b*_*i*_ represents the offset of the visual unit *i*, and *c*_*i*_ represents the offset of the hidden unit *j*. The task of learning RBM is to find the values of these parameters to fit the given training data.

Given a set of randomly selected training data *v*, since the conditional probability value of hidden units only depends on the distribution of explicit units, the conditional probability of hidden units is

(2) $$\begin{array}{c} p\left(h_{j}|v\right)=\sigma \left(\sum_{i=1}^{n}w_{ij}v_{i}+c_{i}\right). \end{array}$$

In the same way, the conditional probability of explicit unit can be easily calculated as follows:

(3) $$\begin{array}{c} p\left(v_{j}|h\right)=\sigma \left(\sum_{j=1}^{m}w_{ij}h_{i}+b_{i}\right). \end{array}$$

*σ*(·) is sigmoid function and is defined as *σ*(*x*)=1/(1+exp(−*x*)). Then, Hinton proposed a contrast diffusion algorithm, which improved the method of obtaining the reconstructed value of the model through a large number of Gibbs. The efficiency of the algorithm is greatly improved, and the updating criteria of weights are as follows:

(4) $$\begin{array}{c} Vw_{ij}=\delta \left({\langle v_{i}h_{j}\rangle }_{\text{data}}-{\langle v_{i}h_{j}\rangle }_{\text{recon}}\right). \end{array}$$

*δ* is the learning rate, 〈·〉_data_ is the expected value of input data, and 〈·〉_recon_ is the expected value of reconstructed data. The above formula shows that the update of weights depends on the difference between input data and reconstructed data, and minimizing this difference can make the hidden layer of RBM better extract the essential features of the input of the explicit layer. By further observing formula (4), it can be found that the training criterion of RBM only needs simple addition and multiplication, so that the calculation amount is not too large, and the weight updating process can be easily completed.

RETRACTED

## 4. Cyclic Neural Network

The ordinary BP network and convolution neural network are both feedforward neural networks. In feedforward neural networks, neurons between layers are connected by edges, while neurons in the same layer are not connected by edges. The neural network is originally constructed by imitating the connection mode of human neurons. In addition, the calculation steps from input to output are also fixed; that is, the number of layers of the network is preset. It is difficult to learn the long-term dependence of input by this connection. In addition, in the language model, the previous text and the current input text are used to predict the next word. Feedforward neural network cannot be completed, but the cyclic network can solve these problems. In RNN, the output of the previous time will also be the input of the current time, so the current output of the network is also related to the input of the previous time, so the operation is to learn the dependency relationship of the sequence.

In theory, RNN can deal with input sequences of any length, but in practice, it is difficult to learn the dependence of sequences due to gradient disappearance or gradient explosion when training networks.  Figure 1 is a structural diagram of a convolutional neural network.

The most basic RNN formula is as follows:

(5) $$\begin{array}{c} h_{t}=f\left(Wx_{t}+Uh_{t-1}+b\right), \end{array}$$

where *x*_*t*_ is the sequence input at time *t*, *W* is the weight matrix between the input layer and hidden layer, and *U* is the weight matrix between neurons in the same hidden layer. *f*(·) is an activation function, generally sigmod, tanh, or ReLU function; *h*_*t*−1_ is the output of the hidden layer at the last moment; *h*_*t*_ is the output of the hidden layer at the current time; and the initial *h*_0_ is generally set to 0.

RETRACTED

Figure 2 is a structure diagram and timing expansion diagram of an RNN.

From the time series expansion diagram of RNN, we can see that the growth of network input will lead to the lengthening of the expanded model. Training networks are basically gradient descent methods, but there is a serious problem in gradient descent methods, which is gradient disappearance or gradient explosion.

## 5. Construction of the Reverse Resource Recovery System of e-Waste Based on DLRNN

### 5.1. Model Hypothesis

The secondary utilization rate and waste rate of electronic waste products, modules, and parts are fixed and known. The unit recovery cost, unit transportation cost, unit inspection, and disassembly cost of electronic waste are fixed and known. The transportation cost in the whole reverse resource network process, including the processing cost of the inspection and reprocessing center, presents a linear relationship. The amount of electronic waste recovered by the recycling center is not specified but varies randomly. The whole reverse resource process only considers the static and single-cycle logistics network.

#### 5.1.1. Reverse Resource Network Model of e-Waste

Profit model of the network: revenue = secondary sales revenue + secondary manufacturing module revenue + secondary manufacturing parts revenue (this formula is not unique), namely,

(6) $$\begin{array}{c} r=\sum_{m}\sum_{k}Y_{km}^{M}qs+\sum_{a}\sum_{n}\sum_{k}Y_{kn}^{\text{NA}}q_{na}^{A}+\sum_{k}\sum_{n}Y_{kn}^{N}q_{nb}^{B}. \end{array}$$

Here, *Y*_*km*_^*M*^ is detecting the number of electronic waste products delivered by the reprocessing center *k* to the secondary consumption market*m*;*qs* is testing the unit product sales price from the reprocessing center *k* to the secondary consumption market *m*; *Y*_*kn*_^NA^ is detecting the number of modules *a* delivered by the reprocessing center *k* to the secondary manufacturing market *n*; *q*_*na*_^*A*^ is the unit sales price of module *a* from detection reprocessing center *k* to secondary manufacturing market *n*; and *q*_*nb*_^*B*^ is the sales price per unit weight of parts *b* from inspection reprocessing center *k* to secondary manufacturing market *n*.

*(1) Carbon Emission Model of Network*. Carbon emission from transportation activities = carbon emission from recycling center to classified storage center + carbon emission from classified storage center to inspection and reprocessing center + carbon emission from inspection and reprocessing center to secondary consumer market + carbon emission from modules transported from inspection and reprocessing center to secondary manufacturing market + carbon emission from parts transported from inspection and reprocessing center to secondary manufacturing market + carbon emission from inspection and reprocessing center to harmless treatment station:

(7) $$\begin{array}{c} t=\sum_{j}\sum_{i}Y_{ij}^{J}W_{s}h_{ij}+\sum_{k}\sum_{j}Y_{jk}^{K}W_{s}h_{jk}+\sum_{m}\sum_{k}Y_{km}^{M}W_{s}h_{km}+\sum_{a}\sum_{n}\sum_{k}Y_{\text{kna}}^{\text{NA}}W_{s}h_{kn}\\ +\sum_{b}\sum_{n}\sum_{k}Y_{\text{knb}}^{\text{NB}}W_{s}h_{kn}+\sum_{k}Y_{k}^{P}W_{s}h_{kp}. \end{array}$$

Here, *Y*_*ij*_^*J*^ is the quantity of electronic waste products delivered by the recycling center *i* to the classified storage center *j*; *W*_*s*_ is carbon emissions per unit distance during transportation; *h*_*ij*_ is the distance from recovery center *i* to the classified storage center*j*; *Y*_*jk*_^*K*^ is the quantity of electronic waste products delivered by the sorting storage center *j*to the detection and reprocessing center *k*; *h*_*jk*_ is the distance from sorting warehouse center*j*to detection reprocessing center *k*; *Y*_*km*_^*M*^ is detecting the quantity of electronic waste products delivered by the reprocessing center *k* to the secondary consumption market *m*; *h*_*km*_ is detecting the distance from the reprocessing center *k* to the secondary consumption market *m*; *Y*_kna_^NA^ is detecting the number of modules *a* delivered by the reprocessing center *k* to the secondary manufacturing market *n*; *h*_*kn*_ is detecting the distance from the reprocessing center *k* to the secondary manufacturing market *n*; *Y*_knb_^NB^ is measuring the number of internal parts *b* delivered by the reprocessing center *k* to the secondary manufacturing market *n*; *Y*_*k*_^*P*^ is detecting that weight of the internal parts of the garbage transport from the reprocessing center to the harmless treatment center; and *h*_*kp*_ is measuring the distance from reprocessing center*k* to harmless treatment center *p*.

RETRACTED

The rule of reverse resource recovery is that the recovery quantity is equal to the classified storage quantity, the recovery quantity is equal to the quantity transported to the inspection reprocessing center, the quantity processed by the inspection reprocessing center is equal to the quantity transported to the secondary consumption market, and the weight of parts is equal.

#### 5.1.2. Long- and Short-Term Memory RNN

The short-term and long-term memory model proposes a new structure called memory cell, and the schematic diagram of the structure is shown in Figure 3. The memory cell consists of four main parts: input gate, self-circulating connected node (self-connected node), forgetting gate, and output gate. It can allow the memory cell to remember or forget its previous state as needed.

The long- and short-term memory RNN (LSTM-RNN) model is different from the standard long- and short-term memory model. In the short-time memory RNN, the starting value of the output gate of a memory cell does not depend on the state value *C*_*t*_ of the memory cell at time step *t*, which enables the network model to perform the calculation of each part more effectively as follows:

(8) $$\begin{array}{c} o_{t}=\sigma \left(W_{o}x_{t}+U_{o}h_{t-1}+b_{o}\right). \end{array}$$

## 6. Result Analysis and Discussion

### 6.1. Model Solution Results

Based on the relevant parameter settings, we use LINGO15.0 × 64 software as a solution tool and use the optimal algorithm of mixed linear programming to solve the problem.

The experimental parameters are substituted into the network optimization model. First, the single-objective optimization is considered separately, that is, the single profit target is maximized (the economic benefit is maximized) and the single-objective carbon emission is minimized (the environmental benefit is maximized). Then, the two-objective model is further optimized, the location change of the detection reprocessing center is obtained, and the location is further optimized. When only a single objective is considered, the optimization results of the network model under the carbon quota policy are shown in Table 1.

According to the above model, because the carbon quota policy sets different carbon emissions, the profit and carbon emissions of the third-party recycling enterprises in the reverse resource network model and the changes of the carbon emissions of the third-party recycling enterprises are shown in Table 2.

From the data in Tables 1 and 2, it can be found that the average profit increased by 1.28%, the average carbon emissions decreased by 4.37%, and the average carbon emissions of third-party recycling enterprises decreased by 12.71% from the original site selection scheme to the current site selection scheme. Under the carbon quota policy, when the carbon emissions allocated to the third-party recycling enterprises change from the original site selection scheme to the current site selection scheme, the profits of the whole reverse resource network show an upward trend. At this time, in order to further reduce the related carbon emissions, the third-party recycling enterprises are required to reduce the total amount of products, modules, and parts that are being tested and reprocessed.

Under the carbon quota policy, when the carbon emissions allocated to the third-party recycling enterprises change from the original site selection scheme to the current site selection scheme, the profits of the whole reverse resource network show an upward trend. At this time, in order to further reduce the related carbon emissions, the third-party recycling enterprises are required to reduce the total amount of products, modules, and parts that are being tested and reprocessed.

RETRACTED

It can be found from Figure 4 that, under the carbon quota policy, with the change of carbon emission quota, compared with the profit of the reverse resource network of the original site selection scheme, the profit of the logistics network of the current site selection scheme has increased a lot, and with the continuous increase of carbon emission quota, its profit has also increased. It can be found that, under the carbon quota policy, the increase of profits is relatively small and the economic benefits are not significant.

It can be found from Figure 5 that, under the carbon quota policy, the carbon emission of the current site selection scheme has been reduced to a certain extent compared with the original site selection scheme. When the carbon emission quota allocated to the third-party recycling enterprises is gradually increased, the carbon emission of the whole logistics network also shows an upward trend, and the reduction of carbon emission is not obvious. In addition, with the gradual increase of carbon emissions of the logistics network, the total carbon emissions of the whole reverse resource recovery network also show an upward trend, and the effect of emission reduction is almost zero.

Through the calculation results of the above network optimization model, it is found that, under the carbon quota policy, the average carbon emissions in the whole reverse resource network activities are reduced by 4.37%. It can be found that, under the carbon quota policy, the carbon emissions are reduced a lot, which has certain environmental benefits.

## 7. Experimental Results and Their Analysis

To show the superiority of the DLRNN in problem classification, compare it with the classical methods that have been proposed. The comparison algorithm mainly consists of two parts, one of which is the recently proposed classic DL algorithm. In order to ensure fairness, the experimental results published by the algorithm are directly quoted. The other part is traditional machine learning algorithms, including classic Naive Bayes and Support Vector Machine.  Table 3 shows the experimental results of problem classification.

Compared with these neural network methods and traditional methods, the experimental results show that DLRNN can handle the problem classification task well. In the TREC dataset, compared with the traditional method DLRNN, it is improved by about 3.5% and, compared with the latest neural network method, it is improved by about 2.4%. In the MSQC dataset, it is improved by about 2.5% compared with the traditional method neural network.

RETRACTED

In order to further analyze the role of each module in the hybrid network framework DLRNN, this section also designed many comparative experiments to verify the effectiveness of each module. In order to ensure the fairness of the comparative experiment, only the tested modules are modified, while the other modules are unchanged. In the contrast experiment, we not only test the function of layering but also compare the layered and nonlayered networks.

Figure 6 shows the test accuracy of the single-layer network and multilayer network in the training process. It can be clearly seen from the experimental results that neither the single-layer convolutional neural network nor the single RNN can achieve the classification accuracy of the hierarchical framework. Among single-layer neural networks, the convolutional network is closest to the classification effect of the hierarchical framework, while RNN is relatively poor. This shows that the convolution network has a strong classification ability. At the same time, extracting text features hierarchically can further improve the ability of problem classification.

Figure 7 shows the test accuracy of the convolution neural network and the nonconvolution neural network in the training process. It can be clearly seen from the experimental results that when CNN in the DLRNN is replaced by any RNN, the classification effect will be seriously reduced. This shows that the convolution network plays an important role in problem classification. In addition, it is found in experiments that if the feature extraction from character to word still adopts a circular network, it will lead to time-consuming training.

Parameter sensitivity analysis: in this paper, the model shows the effects of three superparameters in two datasets Amazon-CDs and Amazon-Books: item embedding dimension *d* and the lengths |*L*| and |*T*| of continuous items of user interaction. The effect of embedding dimension *d* is shown in Figures 8 and 9.

It can be seen from the above figure that when the embedded dimension of the project is too small and the performance of the model recommendation is not good, because the too small dimension of the project is not enough to model the potential features of the project. By increasing the dimension of project embedding, the model has more ability to simulate the complex features of the project. With the increase of project embedding dimension *d*, the performance of the model gradually improves and becomes stable.

RETRACTED

## 8. Conclusion

e-Waste reverse resource recycling system is a comprehensive problem. For the above problems, this paper combines low-carbon theory, carbon footprint calculation theory, low-carbon policy, recycling mode, and network optimization; comprehensively considers qualitative analysis and quantitative analysis; and finally obtains a network model of e-waste reverse resource recycling under the low-carbon policy situation. In this paper, we not only analyze the carbon emissions in the whole transportation process but also the carbon emissions in warehousing, classification, disassembly, handling, and other related activities. The model constructed not only considers the profits of the whole reverse resource network, but also. In this paper, DLRNN is tested on the classic question classification dataset TREC and the dataset MSQC extracted from the question and answer dataset. The experimental results show that DLRNN achieves the best classification results on TREC and MSQC datasets.

## Figures and Tables

**Figure 1:** Structure diagram of the convolutional neural network.

**Figure 2:** Structure diagram and timing expansion diagram of RNN.

**Figure 3:** Memory cell structure diagram of the long- and short-term memory model.

**Figure 4:** Change trend of carbon emission limit to profit.

**Figure 5:** Change trend of carbon emission limit to carbon emission.

**Figure 6:** Comparison of different hierarchical networks on TREC.

**Figure 7:** Comparison of different convolution network modules on TREC.

**Figure 8:** Amazon-CDs.

**Figure 9:** Amazon-Books.

**Table 1:** Single-objective optimization result.

	Profit	Carbon emissions
Profit target alone is the largest	896301.36	255036.61
The single target carbon emission is the smallest	925517.90	201598.07

**Table 2:** Profit, carbon emission, and third-party carbon emission of reverse resource network.

Carbon emission limit	Profit		Carbon emissions		Third-party carbon emissions	
	Original site selection	Current site selection scheme	Original site selection	Current site selection scheme	Original site selection	Current site selection scheme
75000	925617.02	925571.41	232449.62	210147.25	933258.71	708.25
80000	925617.02	933069.07	232449.62	220897.37	933258.71	746.39
85000	925617.02	939249.78	232449.62	222750.21	933258.71	778.92
90000	925617.02	945025.39	232449.62	229749.86	933258.71	849.67

**Table 3:** Result of the DLRNN framework in problem classification.

Classification method	TREC (%)	MSQC (%)
CNN-nonstatic [21]	93.7	—
C-LSTM [22]	94.5	—
DSCNN [23]	95.5	—
CCNN [24]	97.1	—
TF-IDF + SVM	94.6	88.3
DLRNN	98.5	94.7

## Data Availability

The data used to support the findings of this study are available from the corresponding author upon request.
